RETRACTED

# NNK from tobacco smoking enhances pancreatic cancer cell stemness and chemoresistance by creating a β2AR‐Akt feedback loop that activates autophagy

**DOI:** 10.1002/1878-0261.13230

**Published:** 2022-06-05

**Authors:** Xin Chen, Weifan Zhang, Rujuan Liu, Zeen Zhu, Mengyuan Gong, Qiqi Wang, Weikun Qian, Zheng Wu, Qingyong Ma, Zheng Wang

**Affiliations:** ^1^ Department of Otorhinolaryngology Head and Neck Surgery The First Affiliated Hospital of Xi'an Jiaotong University China; ^2^ Department of Hepatobiliary Surgery The First Affiliated Hospital of Xi'an Jiaotong University China

**Keywords:** autophagy, chemoresistance, NNK, pancreatic cancer, stemness

## Abstract

Low responsiveness to chemotherapy is an important cause of poor prognosis in pancreatic cancer. Smoking is a high‐risk factor for pancreatic cancer and cancer resistance to gemcitabine; however, the underlying mechanisms remain unclear. 4‐(methylnitrosamino)‐1‐(3‐pyridyl)‐1‐butanone (NNK) is the main metabolite of tobacco burning and has been shown to be associated with cancer development and chemoresistance. However, in pancreatic cancer, its mechanism remains poorly understood. In this study, we found that NNK promoted stemness and gemcitabine resistance in pancreatic cancer cell lines. Moreover, NNK increased autophagy and elevated the expression levels of the autophagy‐related markers autophagy‐related gene 5 (ATG5), autophagy‐related gene 7 (ATG7), and Beclin1. Furthermore, the results showed that NNK‐promoted stemness and gemcitabine resistance was partially dependent on the role of NNK in cell autophagy, which is mediated by the β2‐adrenergic receptor (β2AR)‐Akt axis. Finally, we proved that NNK intervention could not only activate β2AR, but also increase its expression, making β2AR and Akt form a feedback loop. Overall, these findings show that the NNK‐induced β2AR‐Akt feedback loop promotes stemness and gemcitabine resistance in pancreatic cancer cells.

## Graphical abstract

β2AR, activated by NNK, increases Akt activity and further promotes autophagy, which leads to the formation of stemness and gemcitabine resistance of pancreatic cancer cells. Activation of Akt or downstream signals can increase β2AR expression in a feedback loop.

**Abbreviations**
ATG5: autophagy‐related gene 5
ATG7: autophagy‐related gene 7
cAMP: cyclic adenosine monophosphate
CQ: chloroquine
CSCs: cancer stem cells
EMT: epithelial‐mesenchymal transition
Gem: gemcitabine
NNK: 4‐(methylnitrosamino)‐1‐(3‐pyridyl)‐1‐butanone
PCSCs: pancreatic cancer stem cell spheres
PDAC: pancreatic ductal adenocarcinoma
PI3K: phosphatidylinositol 3‐kinase
PKA: protein kinase A
PKB: protein kinase B
β2AR: β2‐adrenergic receptor

RETRACTED

## 1 Introduction

Pancreatic cancer is one of the most malignant tumors, due to its late diagnosis, aggressive tumor growth, and high level of metastasis, and the overall 5‐year survival rate of patients with pancreatic cancer is less than 10% [1]. Pancreatic ductal adenocarcinoma (PDAC) is the most common pathological type of pancreatic cancer, accounting for more than 90% of cases [2, 3]. Due to the insidious onset, some patients have lost the chance of surgical resection when they are diagnosed, and chemotherapy is the main treatment. Gemcitabine is the most common first‐line chemotherapy drug approved for the treatment of advanced PDAC, either alone or in combination with other chemotherapeutic agents [4, 5]. Although gemcitabine combined with other chemotherapy agents can profoundly improve the prognosis of advanced pancreatic cancer, the development of chemoresistance still leads to poor clinical outcomes [6]. Therefore, it is particularly important to further elucidate the mechanisms of gemcitabine resistance and to find a therapeutic method to reverse it.

Smoking is the first investigated modifiable risk factor for pancreatic cancer development [7]. Epidemiological results show that smokers have a significantly increased risk of developing pancreatic cancer and a worse prognosis than nonsmokers [7]. 4‐(Methylnitrosamino)‐1‐(3‐pyridyl)‐1‐butanone (NNK), a nitrosamine, which is the main metabolite produced by burning tobacco, is thought to have a strong carcinogenic effect [8]. Interestingly, NNK promotes the proliferation [9], migration [10], and stemness [11] of pancreatic cancer cells, and there is a significant correlation between cell stemness and gemcitabine resistance. However, the functional roles and mechanisms of NNK in the sensitivity of pancreatic cancer to gemcitabine treatment remain poorly understood, and thus need to be further clarified.

Autophagy is phagocytosis of cytoplasmic proteins or organelles, which are encapsulated into vesicles and fused with lysosomes to form autophagy lysosomes followed by degradation of encapsulated contents to achieve the metabolic needs of cells and the renewal of some organelles [12]. The process of autophagy can be broken down into five steps: induction, nucleation, elongation, maturation, and degradation. Nucleation of the phagophore occurs following induction by the ULK1/2 complex. Elongation consists of two important processes: ATG12–ATG5‐ATG16L1 complex conjugation and LC3 lipidation to form LC3‐II. Eventually, the isolation membrane is enclosed to form an autophagosome, which will then fuse with the lysosome, forming an autolysosome for degradation. Although the mechanisms of autophagy are not fully understood, studies have shown that it is closely related to chemotherapy resistance [13, 14, 15, 16]. The chloroquine (CQ) autophagy blocker also significantly improves the sensitivity of pancreatic cancer cells to gemcitabine [17].

RETRACTED

Beta‐adrenergic receptor (βAR), a member of the G‐protein‐coupled receptor family, has been paid more attention recently [18, 19]. Three subtypes, β1, β2, and β3, have been identified. βAR is thought to be involved in the biological behaviors of pancreatic cancer, especially β2AR, which mediates chronic stress and its development [9, 20]. In addition, βAR also activates protein kinase B (PKB)/Akt through phosphatidylinositol 3‐kinase (PI3K) and Erk1/2, thereby activating a series of transcription factors to promote the proliferation of pancreatic cancer cells [21, 22].

In this study, we attempted to investigate the contributions and mechanisms of NNK in the resistance of pancreatic cancer cells to gemcitabine. We demonstrated that NNK promotes pancreatic cancer cell resistance to gemcitabine and stemness through increasing autophagic activity, which is mediated by the β2AR‐Akt feedback loop.

## 2 Materials and methods

### 2.1 Cell culture and reagents

The BxPC‐3 and Panc‐1 human pancreatic cancer cell lines were purchased from the Chinese Academy of Sciences Cell Bank of Type Culture Collection (CBTCCCAS, Shanghai, China). The cells were cultured in RPMI‐1640 or DMEM (Gibco, Thermo Fisher Scientific, Waltham, MA, USA) supplemented with 10% fetal bovine serum (FBS) at 37 °C with 5% CO_2_. NNK (1 μm for cells), CQ (10 μm for cells), and gemcitabine (Gem, 5 μm for cells) were purchased from Sigma‐Aldrich (St. Louis, MO, USA), ICI 118551 (10 μm for cells), LY294002 (10 μm for cells) were purchased from MedChem Express (Monmouth Junction, NJ, USA); the inhibitors were dissolved in DMSO according to the manufacturer's protocol.

### 2.2 Colony formation assay and stem cell sphere formation assay

Pancreatic cancer cells were seeded into 6‐well plates at 1000 cells per well for 24 h and treated with different concentrations of drugs for 10 days. Then the 6‐well plates were washed with phosphate‐buffered saline (PBS), fixed with 4% paraformaldehyde, and stained with crystal violet solution for 20 min. The number of colonies was counted in five random fields by microscopy. In addition, after harvesting, resuspension, and counting, 1000 cells were seeded into ultralow attachment 6‐well plates at 1000 cells per well for serum‐free DMEM/F12 medium (containing 20 ng·mL^−1^ EGF, 20 ng·mL^−1^ FGF, and 1% B27) and cultured for 1 week. The number of stem cell spheres was counted under a microscope (Nikon Instruments Inc, Tokyo, Japan).

RETRACTED

### 2.3 siRNA, RNA extraction, and qRT‐PCR

Pancreatic cancer cells were seeded into 6‐well plates 24 h before transfection. siRNA (Gene Pharma, Shanghai, China) and lipofectamine 8000 Transfection Reagent (Invitrogen, Carlsbad, CA, USA) were used according to the manufacturer’s protocols. Total RNA was extracted from cultured pancreatic cancer cells using TRIzol reagent purchased from Invitrogen. cDNA was reverse‐transcribed using a cDNA synthesis kit (TaKaRa, Tokyo, Japan). Quantitative PCR was performed using SYBR qPCR Master Mix (TaKaRa). The mRNA expression level for each sample was determined using the $2^{-\Delta \Delta c_{t}}$ method with three biological replicates for comparative qRT‐PCR.

### 2.4 Immunofluorescence assay

Pancreatic cancer cells were cultivated on circular glass slides in 24‐well dishes after treatment, fixed in 4% paraformaldehyde for 20 min, washed with PBS twice, treated with permeabilization solution (1% Triton X‐100 in PBS), washed with PBS again, and blocked with 5% bovine serum albumin (BSA; Sigma‐Aldrich, Darmstadt, Germany) for 1 h. Samples were incubated with primary antibodies in PBS buffer overnight at 4 °C. Then the samples were washed with PBS twice and incubated with fluorescein isothiocyanate‐conjugated AffiniPure goat anti‐rabbit IgG secondary antibody (dilution, 1 : 300; Beijing Zhongshan Golden Bridge Biotechnology, Beijing, China) for 60 min at room temperature. After the samples were stained with DAPI, images were captured with a ZEISS Instruments confocal microscope (Carl Zeiss, Oberkochen, Germany).

### 2.5 Western blot analysis

Western blot was performed as described previously [23]. Pancreatic cancer cells were seeded in 6‐well plates for 24 h and then treated with various interventions. Then protein lysates were obtained by incubating the cells in RIPA buffer containing proteinase inhibitors for 10 min on ice and centrifugation at 12 000 ***g*** for 15 min at 4 °C. The samples were separated by 10% SDS/PAGE and transferred to PVDF membranes. After blocking with 5% nonfat milk, the membranes were incubated with primary antibodies (LC3, ATG5, ATG7, Beclin1 SOX2, OCT4, Nanog, β1AR, β2AR, Akt, p‐Akt; and β‐actin; all purchased from Cell Signaling Technology, CST, Boston, MA, USA) at 4 °C overnight. Next, the membranes were washed with PBST buffer four times and incubated with peroxidase‐conjugated secondary antibodies for 1 h at room temperature. After washing with PBST buffer four times, the membranes were visualized with an ECL chemiluminescent detection system (Bio‐Rad, Hercules, CA, USA).

### 2.6 Autophagy flux detection

Autophagy flux detection was monitored using three methods in this research: western blot of LC3 (conversion of LC3B I to LC3B II), LC3B punctae immunofluorescence staining and tandem fluorophore detection (Ad‐mRFP‐GFP‐LC3) according to the reported method [24]. Ad‐mRFP‐GFP‐LC3 was purchased from HanBio (Shanghai, China) and the experiment was carried out according to the provided instructions. Cells were plated in 6‐well dishes and were grown to 50% confluence at the time of infection. Then the cells were cultured in DMEM supplemented with 1% FBS and adenoviruses for 2 h at 37 °C. After infection, cells were grown for 48 h in medium with 10% FBS and used for further study. Autophagy was observed under a fluorescence microscope. Autophagic flux was determined by evaluating the number of GFP‐ and RFP‐positive puncta. Owing to the sensitivity of GFP to the acidic environment of autolysosomes, red dots represent autolysosomes and yellow dots represent autophagosomes. The cell autophagy level was qualified by counting red and green dots separately and further analyzed the proportion of autolysosome and autophagosome.

RETRACTED

### 2.7 Statistical analysis

All statistical analyses were performed with graphpad prism 6.0 software (GraphPad, La Jolla, CA, USA). All data are presented as the mean ± SD (standard deviation) of triplicate samples. Differences with a *P* value < 0.05 were statistically significant. Differences between two groups were analyzed by independent sample *t*‐tests, and differences among multiple groups were analyzed by one‐way ANOVA; *P < 0.05, **P < 0.01.

## 3 Results

### 3.1 NNK strengthened stemness and chemoresistance in pancreatic cancer cells

To address the potential role of NNK in pancreatic cancer cells, we first treated BxPC‐3 and Panc‐1 cells with NNK and found that NNK significantly increased the colony formation ability of pancreatic cancer cells (Fig. 1A), which meant that NNK may have a pro‐stemness effect on pancreatic cancer cells. To further confirm this hypothesis, we then examined the effect of NNK on pancreatic cancer spherogenesis, and the results showed that the number of pancreatic cancer stem cell spheres (PCSCs) formed in the NNK‐treated group was significantly higher than that in the control group (Fig. 1B). In addition, the expressions of stem cell markers, OCT‐4, SOX‐2, and Nanog were also enhanced by NNK treatment at both the mRNA and protein levels (Fig. 1C). In summary, the above findings suggested that NNK could strengthen the stemness of pancreatic cancer cells.

**Fig. 1:** NNK strengthens stemness and chemoresistance in pancreatic cancer cells. (A) 1000 pancreatic cancer cells were seeded in a 6‐well plate with or without 1 μm 4‐(methylnitrosamino)‐1‐(3‐pyridyl)‐1‐butanone (NNK) treatment; the cell colony formation assay was performed for 10 days. Representative images are shown (left) and cell colony number was quantified (right; scale bar, 1 cm). Data are presented as mean ± SD of three separate experiments. **P < 0.01 by Student's *t* test. (B) Cells were treated with 1 μm NNK and representative images of the tumor sphere formation assay were captured (left) and sphere number of each group were quantified (right; scale bar, 50 μm). Data are presented as mean ± SD of three separate experiments. **P < 0.01 by Student's *t* test. (C) Panc‐1 and BxPC‐3 cells were treated with 1 μm NNK, western blot (left) and qPCR (right) of indicated markers were performed 48, 24 h later, respectively. Data are presented as mean ± SD of three separate experiments. **P < 0.01 by Student's *t* test. (D) Pancreatic cancer cells (20 000 for Panc‐1, 40 000 for BxPC‐3) were seeded in 12‐well plates and received the indicated treatments. The numbers of cancer cells were counted at the indicated timepoints. Data are presented as mean ± SD of three separate experiments. *P < 0.05; **P < 0.01 by one‐way ANOVA test. (E) 1000 pancreatic cancer cells were seeded in 6‐well plates with or without NNK (1 μm), gemcitabine (gem, 5 μm) treatment; cell colony formation assay was performed for 10 days. Representative images are shown and cell colony number was quantified (scale bar, 1 cm). Data are presented as mean ± SD of three separate experiments. **P < 0.01 by one‐way ANOVA test.

RETRACTED

Increasing evidence suggested that cell stemness is often accompanied by an increase in chemoresistance in pancreatic cancer [25, 26]. Hence, we next aimed to verify whether NNK is associated with gemcitabine resistance in pancreatic cancer cells. Pancreatic cancer proliferation was significantly decreased by gemcitabine, while this phenomenon was partly eliminated by NNK (Fig. 1D). Additionally, using a colony formation assay, we confirmed the above findings (Fig. 1E). In summary, the above findings suggested that NNK could promote the chemoresistance of pancreatic cancer cells.

### 3.2 NNK induced autophagy in pancreatic cancer cells

Notably, the activation of autophagy and related pathways may play an essential role in cancer cell stemness and chemotherapy resistance. Hence, we aimed to determine whether NNK could influence autophagy in pancreatic cancer. We used immunofluorescence to stain LC3 autophagy spots and found that NNK significantly increased the number of LC3 autophagy spots in Panc‐1 cells (Fig. 2A). Moreover, NNK treatment increased LC3B II expression in a time‐ and dose‐dependent manner, which could be enlarged by CQ treatment. P62, an autophagy substrate, protein level was also inhibited by NNK treatment (Fig. 2B and Fig. S1A). To observe the effect of NNK on autophagy more intuitively and accurately, an mRFP‐GFP‐LC3 adenovirus was employed. Owing to the sensitivity of GFP to the acidic environment of autolysosomes, red dots represent autolysosomes, and yellow dots represent autophagosomes [27]. Cells with NNK treatment had more red and green dots compared with the control group (Fig. 2C). Moreover, NNK elevated the autophagolysosome proportion in Panc‐1 cells (Fig. 2C). The expressions of autophagy‐related genes, ATG5, ATG7, and Beclin1 were also enhanced by NNK treatment at both the mRNA and protein levels in a time‐ and dose‐dependent manner (Fig. 2D,E and Fig. S1B,C). We further introduced siRNA targeting ATG5, ATG7, and Beclin1 (Fig. 2F). In response to siRNA treatment, the LC3B II protein level elevated by NNK was significantly decreased (Fig. 2G). The promotion effect of LC3 punctae number by NNK was also inhibited by siATG5, siATG7, and siBeclin1(Fig. 2G and Fig. S1D). Taken together, these results suggested that NNK treatment could influence autophagy in an ATG5‐, ATG7‐, and Beclin1‐dependent way.

RETRACTED

**Fig. 2:** NNK induces autophagy in pancreatic cancer cells. (A) Panc‐1 cells treated with NNK with or without chloroquine (CQ) cotreatment for 24 h; representative immunofluorescence images of LC3 are shown (scale bar, 15 μm). (B) Panc‐1 cells were treated with increasing concentrations of NNK at the indicated timepoints with or without CQ treatment; protein levels were detected using western blot (upper) and quantified (lower). Data are presented as mean ± SD of three separate experiments. *P < 0.05 by one‐way ANOVA test. (C) Cells were transfected with mRFP‐GFP‐LC3 adenovirus, and 48 h later the cells were treated with 1 μm NNK for another 24 h. Cells were then fixed, and the images were captured using a confocal microscope (scale bar, 15 μm; left). Quantification of red and yellow fluorescent dots (middle and right). **P < 0.01 by Student's *t* test. (D) Levels of autophagy‐related gene 5 (ATG5), autophagy‐related gene 7 (ATG7), and Beclin1 in Panc‐1 cells treated with 1 μm NNK for 0, 6, 24 h (left). Levels of ATG5, ATG7, and Beclin1 in Panc‐1 cells treated with the indicated concentrations of NNK for 24 h (right). Data are presented as mean ± SD of three separate experiments. *P < 0.05; **P < 0.01 by one‐way ANOVA test. (E) Western blot to show protein expression of Panc‐1 cells treated with 1 μm NNK at the indicated timepoints (left). Panc‐1 cells were treated with the indicated concentrations of NNK and western blot was performed (right). (F) qRT‐PCR to show the knockdown efficiency in Panc‐1 cells. Data are presented as mean ± SD of three separate experiments. **P < 0.01 by one‐way ANOVA test. (G) Panc‐1 cells were pretreated with the indicated siRNA for 24 h, and then received NNK treatment for an additional 24 h; western blot was performed (left) and immunofluorescence of LC3 were performed, then the LC3 punctae was quantified (right). Data are presented as mean ± SD of three separate experiments. **P < 0.01 by one‐way ANOVA test.

RETRACTED

### 3.3 NNK enhanced the stemness and chemoresistance of pancreatic cancer cells by activating autophagy

The stemness and chemoresistance of cancer cells were reported to be related to cell autophagy [28, 29]. Hence, we tended to determine whether the increase in stemness/chemoresistance of pancreatic cancer cells induced by NNK was due to its effect on cell autophagy. Chloroquine, a classic autophagy inhibitor, was applied in our experiment. It was shown that NNK promoted the colony formation ability in Panc‐1 cells, which could be reversed by CQ cotreatment (Fig. 3A). This result was confirmed by another autophagy inhibitor, autophinib (Fig. 3A). Moreover, the Transwell assay also confirmed similar phenomena in the invasion/migration of Panc‐1 cells (Fig. 3B). The above findings suggested that NNK‐mediated strengthening of stem‐cell‐like behavior in pancreatic cancer cells was autophagy‐dependent. Next, to illustrate the effect of NNK and downstream autophagy in pancreatic cancer cells stemness more directly, we measured the spherogenesis of Panc‐1 cells. The results showed that inhibition of autophagy by CQ or autophinib significantly decreased both the number and size of the tumor sphere in the NNK‐treated group (Fig. 3C and Fig. S1E). Consistently, the upregulation effect of NNK on the expression of cell stemness marker SOX‐2, OCT‐4, and Nanog were also retarded by autophagy inhibition (Fig. 3D and Fig. S1F). In summary, the previous results revealed that NNK enhanced the stemness of pancreatic cancer cells by activating autophagy.

**Fig. 3:** NNK enhances the stemness and chemoresistance of pancreatic cancer cells by activating autophagy. (A) Panc‐1 cells were divided into a control group, NNK (1 μm) group, NNK (1 μm) plus CQ (10 μm) group, and NNK (1 μm) plus Autophinib (10 μm) group. Cells were seeded in 6‐well plates and a cell colony formation assay was performed for 10 days. Representative images are shown (left) and the cell colony number was quantified (right; scale bar, 1 cm). Data are presented as mean ± SD of three separate experiments. *P < 0.05 by one‐way ANOVA test. (B) Panc‐1 cells were treated as in Fig. 3A. Transwell‐based migration (upper) and invasion (lower) assays were performed and quantified (scale bar, 100 μm). Data are presented as mean ± SD of three separate experiments. *P < 0.05 by one‐way ANOVA test. (C) Panc‐1 cells were treated as in Fig. 3A, then stem cell sphere formation assay was performed. Sphere number (left) and diameter (right) were quantified. Data are presented as mean ± SD of three separate experiments. *P < 0.05 by one‐way ANOVA test. (D) qRT‐PCR showing mRNA changes in Panc‐1 cells with indicated treatments for 24 h. Data are presented as mean ± SD of three separate experiments. *P < 0.05 by one‐way ANOVA test. (E) Panc‐1 cells were seeded in 12‐well plates and then received the indicated treatments; cell numbers were counted and analyzed. Data are presented as mean ± SD of three separate experiments. *P < 0.05 by one‐way ANOVA test. (F) 1000 pancreatic cancer cells were seeded in 6‐well plates with the indicated treatments; cell colony formation assay was performed for 10 days. Representative images are shown (left) and cell colony number was quantified (right) (scale bar, 1 cm). Data are presented as mean ± SD of three separate experiments. *P < 0.05 by one‐way ANOVA test.

RETRACTED

We next examined whether NNK‐induced pancreatic cancer chemoresistance was mediated by cell autophagy. A higher number of cells were counted in the NNK cotreatment group compared with the gemcitabine alone group (Fig. 3E and Fig. S1G). However, autophagy inhibition by CQ or autophinib significantly restrained the drug resistance caused by NNK (Fig. 3E and Fig. S1G). The same result was confirmed in the cell colony formation assay (Fig. 3F and Fig. S1H). These findings revealed that NNK enhanced the chemoresistance of pancreatic cancer cells by activating autophagy.

### 3.4 NNK promoted autophagy through the modulation of β2AR and Akt

We previously suggested that NNK is an analogue of catecholamines that can activate βAR efficiently, which prompted us to hypothesize that NNK promoted autophagy by activating the βAR signaling pathway in pancreatic cancer cells. To test this hypothesis, a series of experiments was designed. First, β2AR (the main isoform of βAR expressed in pancreatic cancer) was efficiently knocked down by using a specific siRNA (Fig. 4A). It was shown that NNK intervention had significantly greater LC3 punctae formation compared with the control group, which could be further enlarged by CQ treatment (Fig. 4B and Fig. S1I). In contrast, additional β2AR knockdown had less LC3 punctae formation compared with the NNK group. Chloroquine intervention partially rescued the LC3 punctae formation ability in the NNK plus siβ2AR group, still far less than the NNK plus CQ group (Fig. 4B and Fig. S1I). The promotion effect of NNK on ATG5, ATG7, and Beclin1 mRNA expressions were also inhibited by siβ2AR or ICI 118551, a chemical antagonist of β2AR (Fig. 4C and Fig. S1J). These results indicated that β2AR mediated the promotion effect of NNK on autophagy.

RETRACTED

**Fig. 4:** NNK promotes autophagy by modulating β2AR and Akt. (A) the mRNA (24 h) and protein (48 h) levels of β2‐adrenergic receptor (β2AR) were decreased by siRNA. Data are presented as mean ± SD of three separate experiments. **P < 0.01 by Student's *t* test. (B) Immunofluorescence staining (left) shows LC3 autophagy spots in the control group, NNK group, NNK plus siβ2AR group, NNK plus siβ2AR, and CQ group of Panc‐1 cells, and LC3 punctae was counted and analyzed (right) (scale bar, 15 μm). Data are presented as mean ± SD of three separate experiments. *P < 0.05 by one‐way ANOVA test. (C) The mRNA levels of ATG5, ATG7, and Beclin1 were determined in the control group, NNK group, NNK group, siβ2AR plus NNK group, and ICI118551 plus NNK group. Data are presented as mean ± SD of three separate experiments. **P < 0.01 compared with other groups by one‐way ANOVA test. (D) Panc‐1 cells were pretreated with LY294002 (10 μm) or CQ (10 μm), then received NNK (1 μm) treatment for 24 h. LC3 punctae was counted and analyzed by immunofluorescence microscopy. Data are presented as mean ± SD of three separate experiments. *P < 0.05 by one‐way ANOVA test. (E) Western blot to show LC3 protein change in each group of Panc‐1 cells 24 h after treatment. (F) qRT‐PCR showing mRNA changes in Panc‐1 cells 24 h after receiving the indicated treatments. Data are presented as mean ± SD of three separate experiments. **P < 0.01 compared with other groups by one‐way ANOVA test.

As a G‐protein‐coupled receptor embedded the cell membrane, βAR senses the stimulation of extracellular ligands such as NNK and transduction signals through various intracellular pathways. Previous reports showed that NNK could activate Akt signaling [30]. Hence, we introduced a chemical inhibitor of Akt, LY294002, for further experiment. As we can see, additional LY294002 intervention showed less LC3 punctae formation upon NNK treatment, suggesting that Akt signaling may be an important mediator of NNK‐induced autophagy (Fig. 4D and Fig. S1K). To further test the role of Akt signaling in our experiment, we used siAkt to repeat our experiment. In response to Akt siRNA treatment in Panc‐1 cells, LC3B II turnover caused by NNK was significantly reduced (Fig. 4E). Furthermore, the mRNA levels of ATG5, ATG7, and Beclin1 were also decreased upon Akt signaling inhibition (Fig. 4F). Taken together, these results suggested that NNK could promote cell autophagy through partial Akt signaling.

RETRACTED

### 3.5 NNK formed a potential β2AR‐Akt feedback loop in pancreatic cancer cells autophagy

The above findings suggested that the autophagy‐promoting effect of NNK was β2AR‐ and Akt‐dependent. Next, clearly elucidating the up‐ and downstream relationship between β2AR‐Akt and NNK‐induced pancreatic cancer cells autophagy was critical to our research. In general, membrane receptors are the initiators of signaling pathways when the cell is externally stimulated. Hence, we hypothesized that Akt may be a downstream target of β2AR. To test this, we first aimed to exclude the influence of β1AR on NNK‐induced pancreatic cancer βAR activation, and the results showed that β1AR knockdown (Fig. 5A) had no effect on the activation of Akt (Fig. 5B); however, β2AR knockdown and inhibition significantly suppressed Akt activation (phosphorylation) and LC3 maturation (Fig. 5B,C), which suggested that the β2AR‐Akt axis was the main pancreatic cancer cells autophagy inducer after NNK stimulation. However, we accidentally discovered that β2AR expression was influenced by NNK in pancreatic cancer cells (Fig. 5C), which reminded us that there may be a potential β2AR‐Akt‐autophagy feedback loop underlying the effects of NNK. To explore this hypothesis, we treated Panc‐1 and BxPC‐3 cells with NNK for different time periods and found that the expression of β2AR (rather than β1AR) was increased in a time‐dependent manner (Fig. 5D), and this trend can be blocked by inhibitors (Fig. 5E). Moreover, at the protein level, NNK also promoted β2AR expression and Akt activation (Fig. 5F). In conclusion, these findings suggested that NNK activated autophagy through the β2AR‐Akt pathway and increased β2AR expression levels to further strengthen this autophagy activation process, thus forming a potential β2AR‐Akt feedback loop in pancreatic cancer cells autophagy.

**Fig. 5:** NNK forms a potential β2AR‐Akt feedback loop in pancreatic cancer cells autophagy. (A) The mRNA and protein levels of β1‐adrenergic receptor (β1AR) were decreased by siRNA. Data are presented as mean ± SD of three separate experiments. **P < 0.01 by Student's *t* test. (B) Western blot assay to detect indicated proteins when cells treated with siβ1AR or siβ2AR 24 h after treatment. (C) Panc‐1 cells were pretreated with siβ2AR, ICI118551 (10 μm), CQ (10 μm), then received NNK (1 μm) treatment for 24 h, and immunoblotting was performed. (D) Panc‐1 (upper) and BxPC‐3 (lower) cells were treated with NNK (1 μm) for the indicated hours and cell total RNA was extracted. qRT‐PCR was performed to examine the mRNA levels of β1AR and β2AR. Data are presented as mean ± SD of three separate experiments. * *p* < 0.05; **P < 0.01 compared with the control group by one‐way ANOVA test. (E) Relative protein levels of β2AR when cells were treated with NNK or ICI 118551. Data are presented as mean ± SD of three separate experiments. *P < 0.05 by one‐way ANOVA test. (F) Western blot to show protein expression levels when cells received NNK treatment at the indicated timepoints.

RETRACTED

## 4 Discussion

Pancreatic cancer is one of the most lethal malignancies, with a 5‐year survival rate of less than 10% [1]. The incidence of pancreatic cancer is increasing each year, but due to late diagnosis and the rapid progression of the disease, only a small number of patients can receive radical excision after a clear diagnosis [31]. Chemotherapy is also a treatment for patients with advanced pancreatic cancer, and drugs such as gemcitabine are first‐line effective treatments in management. Gemcitabine was approved for clinical use in 1995 by inhibiting DNA synthesis and blocking the progression of the G1/S stage of the cell cycle [32]. Clinically, gemcitabine resistance often occurs, leading to failure of first‐line chemotherapy. Therefore, it is important to explore the mechanism of gemcitabine resistance. NNK is one of the byproducts of burning tobacco and has been reported to be related to drug resistance against various chemotherapeutic drugs [33, 34]. Cancer stem cells (CSCs) are closely related to the generation of drug resistance, their self‐renewal function, formation/maintenance of the CSCs phenotype, and cytoprotective machinery, allowing CSCs to survive after drug exposure. Moreover, autophagy has been shown to play an important role in many biological properties of pancreatic cancer cells, including survival, dormancy and epithelial‐mesenchymal transition (EMT), metastasis, and gemcitabine resistance [35]. However, the relationship between NNK, autophagy, stemness, and gemcitabine resistance in pancreatic cancer remains unclear.

Therefore, in the present study we aimed to determine the effect of NNK on stemness and gemcitabine resistance. First, we used the Panc‐1 and BxPC‐3 pancreatic cancer lines for our experiments and demonstrated that NNK promoted cell growth and sphere formation. Moreover, NNK increased the expression levels of OCT‐4, SOX‐2, and Nanog, which were thought to play an important role in tumor stem cells. It is consistent with previous research that elevated levels may indicate increased stemness in tumor cells [35, 36, 37, 38]. As described in other tumors, NNK promotes tumor progression, including proliferation, invasion, stemness, and drug resistance [39], our experiments also confirmed that NNK can enhance its progression. Interestingly, NNK may promote both stemness and gemcitabine resistance, which was ultimately seen as a challenge for pancreatic cancer treatment. Since LC3 and p62 detection has become an acceptable method for monitoring autophagy and autophagy‐related processes [40, 41], our results showed that NNK can change the expression of LC3 and p62, which indicated that NNK can indeed promote the production of autophagy. We further confirmed that NNK promoted the expression of ATG5, ATG7, and Beclin1, and after knockdown of these autophagy‐related genes, LC3 expression also changed accordingly. Thus, we hypothesized that NNK promoted stemness and gemcitabine resistance in pancreatic cancer cells by activating autophagy. We confirmed this through conducting experiments with CQ [42]. As a lysosomal inhibitor, CQ was commonly used to block autophagy, which assumed that it primarily blocks lysosomal degradation. Additionally, CQ was proved to inhibit autophagy mainly by impairing the fusion between autophagosomes and lysosomes, without substantially decreasing the acidity and degradative activity of lysosome [42]. Moreover, CQ induced an autophagy‐independent severe disorganization of the Golgi and endo‐lysosomal systems. In addition, CQ treatment disorganized the Golgi complex and the endo‐lysosomal system in an autophagy‐independent way [42]. Hence, we applied another autophagy inhibitor, autophinib, and got a similar result as CQ treatment. Therefore, studies on autophagy disorders caused by tobacco metabolites can be confirmed, and this phenomenon also exists in other tumors [43, 44].

RETRACTED

Finally, we tried to determine the molecular mechanism by which NNK promotes autophagy. βAR is a member of the G‐protein‐coupled receptor family, and intracellular signaling after βAR activation is largely modulated through cyclic adenosine monophosphate (cAMP) and protein kinase A (PKA), triggering the activation of a series of transcription factors and promoting the expression of related genes [45]. Several studies have shown that βAR is closely related to autophagy, but whether it promotes or inhibits autophagy is not completely consistent across studies [46, 47, 48]. NNK is a βAR agonist [49], and our experiments demonstrate that NNK activated autophagy through β2AR but not β1AR. Studies have shown that NNK could activate Akt, Erk1/2 signaling [50, 51]. Our previous research also revealed that HIFα may be a potential target for NNK [52]. Akt and Erk1/2 signaling were two classical pathways reported to be associated with cell autophagy. Hence, we mainly focused on these two signalings and we found that NNK regulated Akt via β2AR in different pancreatic cancer cells. β2AR/Akt inhibition partially inhibited NNK‐induced autophagy. Moreover, we also found that this process can increase the expression of β2AR, further enhancing autophagy. Normally, NNK acts as an activator of β2AR, but does not increase the expression of β2AR. But the specific step that increased β2AR protein expression remains to be confirmed by further experiments.

RETRACTED

## 5 Conclusion

In summary, we discovered that NNK promotes human pancreatic cancer stemness and gemcitabine resistance. We also demonstrated the mechanism by which NNK regulated the β2AR‐Akt feedback loop, which activated autophagy. This may explain the mechanism by which smoking promotes gemcitabine resistance (Fig. 6), but further mechanisms should be explored.

**Fig. 6:** Proposed working model of NNK in pancreatic cancer. β2AR, activated by NNK, increase the Akt activity and further promote autophagy, which leads to the formation of stemness and gemcitabine resistance of pancreatic cancer cells. Activation of Akt or downstream signals can increase β2AR expression in a feedback loop.

## Conflict of interest

The authors declare no conflicts of interest.

## Author contributions

XC and WZ performed most of the experiments, treated data, and wrote the article; RL, MG, ZZ, and QW participated in analyzing the data and organized the figures; WQ and ZWu read and reviewed the article. ZWa and QM designed the experiment and article. All authors read and approved the final article.

## Consent for publication

We obtained consent to publish from the participants to report individual data.

## Supporting information


**Fig. S1.** NNK promotes the malignant behavior of BxPC‐3 cells via autophagy induction through β2AR signaling.

## Data Availability

All data generated or analyzed during this study are available from the corresponding author on reasonable request.
